The article "The Use of a Hypoallergenic Dermal Matrix for Wrapping in Peripheral Nerve Lesions Regeneration: Functional and Quantitative Morphological Analysis in an Experimental Animal Model" was retracted in 2024. Reasons: signs of a paper mill; suspected computer-generated content; unreliable results or conclusions; concerns about the data.

# The Use of a Hypoallergenic Dermal Matrix for Wrapping in Peripheral Nerve Lesions Regeneration: Functional and Quantitative Morphological Analysis in an Experimental Animal Model

**DOI:** 10.1155/2019/4750624

**Published:** 2019-06-17

**Authors:** Michele Rosario Colonna, Antonina Fazio, Alfio Luca Costa, Franco Galletti, Roberto Lo Giudice, Bruno Galletti, Cosimo Galletti, Giorgio Lo Giudice, Giovanni Dell'Aversana Orabona, Igor Papalia, Giulia Ronchi, Stefano Geuna

**Affiliations:** ^1^Department of Human Pathology, University of Messina, Italy; ^2^Department of Clinical and Experimental Medicine, University of Messina, Italy; ^3^School of Dentistry, University of Barcelona, Spain; ^4^Department of Maxillofacial Surgery, School of Medicine, University of Naples “Federico II”, Italy; ^5^Biomedical and Dental Sciences and Morphofunctional Imaging, University of Messina, Italy; ^6^Department of Clinical and Biological Sciences, University of Turin, Italy

## Abstract

**Introduction:**

The aim of this research was to test, in an animal model, the nerve regeneration technique with a hypoallergenic acellular dermal matrix used to wrap the microsurgical neural suture.

**Materials and Methods:**

Two groups of rats received the cut of limb right median nerves. The regeneration technique considers for both groups an end-to-end nerve suture. In the experimental group (A) was used also a wrapping protocol by a conduit of collagen matrix currently used in oral surgery. The animals underwent functional grasping tests (at 1, 3, 5, and 7 months) and a histological and quantitative analysis of distal nerve was performed at the end of experimental time.

**Result:**

After seven months, the grasping test reveals functional recovery in each tested animal; this improvement is more evident in Group A. The fibers appear well organized with restored myelin sheaths in both groups. Group A showed a great quantity of connective tissue surrounding the nerve. The quantitative morphology analysis in both groups shows a similar fibers density, fiber diameter, and myelin thickness. The differences between the groups in axon mean diameter are significant. In Group A M/d, D/d, and g-ratio is significantly higher compared to control group.

**Conclusions:**

Histological and functional assessments show a functional recovery of the injured nerve in the test groups, stressed by the results of the grasping tests and the meaningful increasing in fiber diameter and higher g-ratio. Moreover, a connective tissue cuff distinguishes the distal portion of the injured nerve. Considering the easy availability and handling of the material used in this study we can conclude that this experimental technique can be considered as a valid alternative to protect nerves in nerve wrap surgery.

## 1. Introduction

In plastic, otolaryngology, oral, and maxillofacial surgery, nerve repair is required when, for traumatic events, malformations, or oncological diseases, a nerve lesion occurs [1, 2].

The most frequent peripheral nerve injuries are caused by upper limb traumas. Also, craniofacial soft tissue injuries, isolated or in combination, can determinate nerve lesions [3, 4].

The facial nerve trauma causes are classified into accidental and surgical (unavoidable or iatrogenic) [5].

Kretlow et al. report that these injuries are the most common traumatic craniofacial damage (10% of all emergencies) and determine facial palsy stands between 5 and 25% [6].

During craniofacial surgery (pontocerebellar, parotid, and temporal bone) a facial nerve trauma may occur. In 7%-10% of temporal bone fractures facial nerve pathology is present [7].

In pediatric and geriatric patients slips, trips, and falls are the main cause of facial traumas, while violence and motor vehicle accidents are predominant in adults [6, 8, 9].

Loss of sensory and motor function in the anatomic innervated area or development of neuropathic pain is pathognomonic symptoms [10].

A neurorrhaphy is recommended when the nerve recovery does not occur due to nerve gap, neuroma, and scar tissue formation. The objective is to obtain the axons regeneration with minimal loss of fibers at the suture line [11].

Several studies have been carried out to identify the gold standards in the surgery approach of nerve repair according to the different clinical situations to be treated: sutures, glues, grafts, or tubules were considered.

Some surgeons prefer to use collagen sleeves or fibrin glue for facial nerve repair [12].

The clinical observation shows how the best results are achieved when the surgical technique is tensionless, performed with few stitches put in the outset connective sheath. Nerve trunk dissection should be avoided, delicate perineural tissue manipulation is needed, and nerve gaps more than 20 mm require a nerve graft to be repaired [13–17].

However, complications like nerve scarring and neuroma may occur, causing the failure of regenerative procedures in peripheral nerve surgery [13–17].

Latest generation glues can be used as an alternative to sutures, especially in the case of smaller trunk repair. In order to avoid sacrifice of nerves used as grafts, tubules in synthetic materials or autogenous conduits (arteries, veins) can be used [18–20].

In order to maintain distal effector function in case of more proximal trunk lesion some surgical, selective procedures as babysitting and nerve transfers have also been proposed [21].

In this animal model study, a collagen substitute as an alternative for nerve wrapping and repair was tested.

## 2. Materials and Methods

For the study were selected 16 Wistar adult female rats weighing between 200 and 300 g.

Experimental surgery was carried out at the Microsurgical Laboratory of the Ecole de Chirurgie in Paris (Institutional license from the “Direction Départementale de la Protection des Populations,” DDPP number C-75-05-23) according to the French law on experimental animal research (law no. 87– 848, October 19, 1987). All the surgeries were carried out by expert surgeons certified by the “Service Protection et Santé Animals du Ministère de l'Agriculture.”

The animals, caged separately under a normal light cycle and fed* ad libitum*, were numbered with the international classification and divided into two groups of eight animals (A, B).

8-12 hours before surgery a period of fasting was observed; a suspension of fluid intake for 2-4 hours before anesthesia was practiced. Anesthesia was achieved with intraperitoneal tiletamine and zolazepam (3mg/Kg) and the dissection performed under magnification (2,5-0,4 x Leica microscopes)

The upper arm and axillary region were then shaved and cleansed with antiseptic solution; an incision was performed following the margin of pectoralis muscles to expose the brachial plexus in the axilla.

On the left arm, the median nerve was then identified and transected with a razor before its division into the terminal branches. On the right side, the procedure was repeated, and the proximal stump buried with 7/0 sutures in a subpectoral muscle pocket. Median nerve burying was performed to prevent spontaneous reinnervation, which could produce interference in functional tests. This modification would allow a greater stability in the nontreated median nerve limb and therefore a better evaluation of the functional recovery of the contralateral nerve repair if it occurred.

Different procedures were then applied to each test side (left arm). In Group A, a direct end-to-end suture was performed and a collagen sheath derived from an acellular hypoallergenic dermal matrix (ADM) (OrACELL®), used in dentistry, that retains native growth factors, collagen, and elastin was wrapped around the suture into a protective sleeve 10 mm long (5 mm from each side from the suture). 9/0 nylon sutures were used [23, 24].

In Group B (control) an end-to-end nerve suture was performed. The wounds of surgical accesses were sutured in Nylon 3/0.

After surgery each animal was caged separately and fed* ad libitum*, constantly followed and monitored in consultation with the central veterinary service and, if necessary, treated with analgesics (carprofen sub cut. 4-5 mg/kg once or twice/day).

In both groups, the functional effects of the therapy have been monitored by the modified grasping test shown by Papalia et al., in order to avoid the limitations that occur using the classical grasping test device such as the tendency of test animals to walk on the grid and the wrist flexion while holding the grid bars. [25] At the end of the observation time (7 months), the rats were sacrificed with an intraperitoneal anesthetic overdose and a histologic analysis of the treated area was performed.

### 2.1. Functional Analysis

During the postoperative period, all animals were tested for flexor digitorum muscle function using the grasping test, from the first month (T_1_) and then every 2 months (T_2_, T_3_), until the sacrifice (T_4_) [25, 26]. For measurement the dynamometer (BS-GRIP Grip Meter- 2 biological Instruments, Varese, Italy), consisting of a precision balance connected to a grid for the animal to grasp, was used.

The test was performed by holding the rat by the tail and bringing it closer to the grid allowing it to grasp and pull. The value recorded was the maximum weight that the animal pulled to maintain its grip before loosening it. For each group numerical data detected from T_1_ to T_4_ are expressed as mean and standard deviation. (SD).

The difference of rat grip force between groups, in each observation time, was statistically assessed. P<0,05 was considered statistically significant (Table 1, Figure 1).

### 2.2. Histology and Quantitative Analysis

Distally to the repair site, a 20 mm segment of left median nerve was taken, including in Group A the collagen wrapping.

The samples were immediately fixed in glutaraldehyde 2.5% in 0.1M PBS (pH 7.4) for five-six hours. Following postfixation in osmium tetroxide 2% for two hours they were dehydrated in ethanol (from 30% to 100%).

The samples were then washed in propylene oxide and embedded in resin (equal parts of Araldite M and Harter, which contained 0.5% of dibutyl phthalate plasticizer and 1-2% of accelerator 964).

For high-resolution optical microscopy, semithin transversal (thickness=2.5 *μ*m) sections were cut, starting from the distal stump of each sample, using an Ultracut UCT ultramicrotome (Leica Microsystems). Sections were stained with toluidine blue (1%) and analyzed with a DM4000B microscope equipped with digital camera DFC320 and IMG50 Image Manager System (Leica).

One section for each animal sample was randomly chosen and the cross-sectional area was examined (Figures 3-4).

Then, 14 fields in each section were selected using a systematic random sampling protocol for stereological and morphometrical analysis.

To avoid edge effect and distortions, a procedure with two-dimensional dissector based on the choice of the fibers in sections upper part, was applied.

For each observation field (Oa) randomly selected, the number of fibers (Nf) was manually counted and their density/mm^2^ (De) was calculated according to the size of the observation field (De=Nf x1000/Oa) (Table 2).

The areas of fibers and axons were measured, allowing the calculation of internal diameter of myelin = axon diameter (d) and external diameter of myelin = fiber diameter (D) and myelin thickness (M) as well the ratio M/d; D/d; and d/D (g-ratio) was calculated [22] (Table 2, Figure 2).

Then for each sample and for the two groups means and SD of quantitative parameter was made, and data were analyzed. The differences for values of P<0,05 were considered statistically significative.

Both statistical analyses were performed using SPSS 17.0 for Window package and Platform Prism Software package (GraphPad, La Jolla, CA, USA).

## 3. Results and Discussion

### 3.1. Results

#### 3.1.1. Functional Analysis

The grasping test result in each group of rats shows that to maintain its grip in T_0_, Group A rats exert an inferior average strength compared to the one registered in Group B (18,5± 30,32 grams vs. 33±20,28 grams). No grip is shown in 63,5% of first group test animals versus 12% of control group.

In T_1_ and T_2_ Group A test animals exert superior average strength compared to Group B (112,5±33,32 grams vs. 102,37±40,44 grams and 144,75±50,33 grams vs. 146,75±31,24 grams). In T_1_ only one test animal keeps exerting force=0. From T_2_ is registered a functional recovery in every test animal. In T_3_ the results show a greater ability to exert force in Group A. The difference between the two experimental groups is not statistically significant.

#### 3.1.2. Histology and Quantitative Analysis

The histological observations of the samples seem substantially analogues. The myelinated fibers appear well-organized with regenerated myelin sheaths. The experimental Group A showed a great quantity of connective tissue surrounding the nerve, which is not present in control group. Grafting area in Group B did not show any immunological response or chronic inflammation of nervous and connective tissues (Figures 3 and 4).

The quantitative morphologic analysis in cross-sectional area shows in both groups a similar fiber density (38653±7184 N/mm^2^ vs. 40972±4287 N/mm^2^). Differences between the groups in axon mean diameter (d) (2,68±0,42 *μ*m vs. 37±0,16 *μ*m) is significant (p<0,05)

Fiber diameter and myelin thickness are almost comparable in wrapped nerves than in simple repair (3,62±0,59 *μ*m - 0,47±0,09 *μ*m vs. - 3,37±0,19 *μ*m - 0,50±0,03 *μ*m).

M/d, D/d ratio in the two groups are, respectively: 0,19±0,01 1,38±0,02 and 0,23±0,02 1,46±0,04. The differences are highly significant (p<0,01) [Table 2]

In Group A g-ratio (0,73 ±0,01) is higher than the one identified in Group B (0, 69±0,02). The statistical analysis shows differences highly significant (p<0,01)

### 3.2. Discussion

In every district the spontaneous nerve recovery is a physiological possibility subsequent a nerve interruption [27].

Millesi et al. showed that peripheral nerves are considered as gliding structures, made up and surrounded by proper connective tissues themselves capable of gliding [13–17].

When natural healing is not possible the main objective of nerve repair techniques is regenerating sensory, motor, and autonomic axons with limited loss of fibers among the suture line [11].

The wrapping with different materials, whether autologous or heterologous, has been introduced to facilitate nerve repair processes; tubules constitute a regrowth protection and stimulation [18–20, 28].

Some materials were identified as possible wrapping for nerve repair, and collagen has shown the best result for hits biocompatibility and adaptability [18, 20].

The use of collagen conduits could be also considered when complex surgical procedures are planned. Therefore, the wrapping/tubulization of long nerve grafts (whether auto or allografts), such as in cross facial nerve grafting, with collagen or collagen/GAG conduits, could be suggested.

Since collagen has also been successfully used as a conduit for nerve regeneration, for short gaps (no more than 3-4 cm) proximal and distal stump coaptation into a collagen tube, it could also be considered as a valid alternative to autologous vein (filled by free muscle or not) [18].

The animal model used by the authors has been the simulation of an upper limb nerve lesion and surgical therapy. This procedure can be considered a standard in research of nerve regeneration, furthermore, allowing functional assessment [29].

Histological results of our research show how the use of ADM in guided bone regeneration and oral soft tissue correction does not modify the injured nerve healing. This is stressed by the presence of well-organized myelinated fibers in the distal stump of the nerve and no significant difference in fiber density and myelin thickness between the two groups [30, 31].

The morphological evidence of the matrix action is shown by the presence of a connective tissue and collagen cuff around the graft area, as more clearly highlighted in Group A observations. No immunological or inflammatory response vs. the dermal matrix was observed.

A soft, tensionless repair can recreate the gliding apparatus described by Millesi allowing nerves to have their own range of free motion [14–17].

The grasping test progression in time highlights in an initial phase a slow pace in the functional recovery process; this is stressed in T1 by favorable results in the control group in both the number of test animals capable of exert force and the entity of the aforesaid force. In further controls; every test animal shows a grasping ability with progressively overlapping exerted force values. Seven months after the procedure, the functional analysis shows a superior strength exerted by the rats subjected to the tubulization procedure compared to the group in which the end-to-end anastomosis was not protected, although the data are not statistically significant. Moreover, the conductive ability of the nerves is objectified by the significant increase in fiber diameter since this dimension is proportional to the conduction velocity space constant and the wavelength of the nerve impulse. The same assessment is highlighted by the higher g-ratio identified in Group A compared to the control group that analyses the perineuronal myelin quota and subsequently the jumping conduction potential binds to the action of Schwann cells [32].

Native growth factors present in ADM components as mediators for Schwann cells proliferation and reorganization of molecular and ionic pattern in regenerating nerve sheaths could explicate how these conduits enhance fiber regeneration [23]

Collagen properties in protection against scar through a reduction of TGF beta and other proinflammatory cytokines might play a role in creating a favorable environment for nerve regeneration [23, 30].

The overall assessment of anatomical and functional tests shows the efficacy of our technique. The dermal matrix use shortens the surgical times, avoiding the harvest of conduits from different donor sites. The thick collagen fiber layer observed around the nerve can be an effect of the grow factors contained in the matrix itself. Considering that the dermal matrix use has no adverse effect, we believe that the technique is ready for a clinical application.

## 4. Conclusions

The collagen membrane tested has never been proposed in conventional tubulisation techniques for nerve repair.

In this animal model study, the use of AMD induced in some aspects a better recovery in neuronal activity.

In the light of the experimental evidence we can conclude that this experimented technique allows, same as others, an efficient nerve trunk repair. The collagen conduit, after clinical trial, can be considered as an alternative to generally used nerve wrap materials to protect nerve repair and its use could be extended to all peripheral nerve surgery. The advantages are the easy availability and handling of the material used and the simplification of the surgical technique since the harvesting of arteries or veins in a different surgical site, in accordance with some nerve wrapping techniques, is avoided.

## Figures and Tables

**Figure 1:** Grasping test results (grams) at T1 - T4 (T_1_ = 1 month, T_2_ = 3 months, T_3_ = 5 months, and T_4_ = 7 months).

**Figure 2:** Histograms showing the morphoquantitative analysis of the regenerated myelinated fibers after 7 months from the surgery of Group A (end-to-end suture with a conduit of collagen matrix - OrACELL® - wrapped around the suture into a protective sleeve) and Group B (end-to-end suture only). Values in the graphics are expressed as mean + SD. P>005 (**∗** = statistically significant value).

**Figure 3:** Representative low-magnification (8x) images of toluidine-blue stained semithin transverse sections of regenerated median nerve repaired with end-to-end nerve suture, with (Group A) or without (Group B) a conduit of collagen matrix (OrACELL®) wrapped around the suture into a protective sleeve. Seven months after surgery, the presence of the collagen layer (C) around the suture zone is still visible in Group A. BAR=500*μ*m.

**Figure 4:** Representative high-resolution (40x) light microscopy images of toluidine-blue stained semithin transverse sections of regenerated median nerve repaired with end-to-end nerve suture, with (Group A) or without (Group B) a conduit of collagen matrix (OrACELL®) wrapped around the suture into a protective sleeve. Seven months after surgery, in both groups, regrowing myelinated fibers (F) with well-organized myelin sheaths (M) are detected. BAR=20*μ*m.

**Table 1:** Groups A and B grasping test results (grams). Functional results at T_1_ - T_4_ (T_1_ = 1 month, T_2_ = 3 months, T_3_ = 5 months, and T_4_ = 7 months).

	Group A				Group B			
	T_1_	T_2_	T_3_	T_4_	T_1_	T_2_	T_3_	T_4_
1	0	90	77	245	32	130	200	224

2	0	110	135	278	0	133	112	100

3	14	82	152	248	20	134	135	170

4	0	100	195	238	70	142	180	200

5	0	80	72	90	40	82	125	224

6	66	126	142	226	34	106	166	208

7	0	132	210	270	24	60	128	202

8	68	180	175	254	44	32	128	186

Average	18,5	112,5	144,75	231,125	33	102,375	146,75	189,25

sd	30,32	33,32	50,33	59,4	20,28	40,44	31,24	40,34

**Table 2:** Quantitative analysis data: average and sd in each sample and in Groups A, B of Axon diameter (d), fibre diameter (D), myelin thickness (M)(*µ*m), and M/d; D/d; and d/D ratio.

	Group A							Group B						
	Density	Axon Diameter (d)	Fiber Diameter (D)	Myelin thickness (M)	M/d	D/d	d/D (g-ratio)	Density	Axon Diameter (d)	Fiber Diameter (D)	Myelin thickness (M)	M/d	D/d	d/D (g-ratio)
1	33317	2,86	3,87	0,50	0,19	1,38	0,74	39519	2,49	3,47	0,49	0,21	1,42	0,71

sd	7440	1,44	1,77	0,23	0,08	0,16	0,1	10478	0,92	1,14	0,16	0,05	0,11	0,06

2	3931	2,53	3,43	0,45	0,19	1,38	0,73	43631	2,31	3,32	0,51	0,23	1,45	0,69

sd	9487	1,09	1,29	0,13	0,05	0,11	0,05	9476	0,88	1,14	0,17	0,06	0,11	0,05

3	49522	2,37	3,21	0,42	0,19	1,38	0,73	46178	2,36	3,25	0,44	0,20	1,41	0,72

sd	12800	0,89	1,06	0,12	0,06	0,11	0,06	9438	0,98	1,18	0,13	0,06	0,12	0,06

4	34597	2,82	3,69	0,43	0,17	1,34	0,75	39968	2,57	3,63	0,53	0,23	1,45	0,70

sd	9076	1,19	1,37	0,12	0,05	0,10	0,06	12026	1,09	1,36	0,17	0,08	0,16	0,07

5	42993	2,26	3,08	0,41	0,20	1,40	0,72	31847	2,58	3,63	0,53	0,22	1,45	0,70

sd	11114	1,07	1,25	0,12	0,06	0,12	0,06	7626	1,10	1,34	0,16	0,07	0,13	0,06

6	38216	2,90	3,93	0,51	0,19	1,38	0,73	43631	2,15	3,09	0,47	0,24	1,48	0,68

sd	6369	1,02	1,24	0,15	0,05	0,11	0,05	7050	0,93	1,12	0,14	0,08	0,16	0,07

7	44585	2,23	2,94	0,36	0,18	1,35	0,75	41998	2,23	3,24	0,51	0,25	1,50	0,67

sd	10070	1,04	1,20	0,11	0,05	0,11	0,06	9391	0,93	1,14	0,15	0,09	0,19	0,07

8	26671	3,47	4,77	0,65	0,20	1,41	0,72	41003	2,28	3,34	0,53	0,26	1,53	0,66

sd	8494	1,54	1,89	0,21	0,06	0,13	0,06	12190	1,16	1,43	0,17	0,10	0,20	0,08

AVERAGE	38652	2,68	3,62	0,47	0,19	1,38	0,73	40972	2,37	3,37	0,50	0,23	1,46	0,69

SD	7184	0,42	0,59	0,09	0,01	0,02	0,01	4287	0,16	0,19	0,03	0,02	0,04	0,02

## Data Availability

The data of grasping test results used to support the findings of this study are available from the corresponding author upon request.
